# 3D High-Frequency Ultrasound Imaging of Cartilage-Bone Interface Compared with Micro-CT

**DOI:** 10.1155/2020/6906148

**Published:** 2020-05-31

**Authors:** Yanping Huang, Choi Han Chan, Guangquan Zhou, Yongping Zheng, Chun Hoi Yan, Chunyi Wen

**Affiliations:** ^1^School of Physics and Optoelectronic Engineering, Foshan University, Foshan, Guangdong, China; ^2^Department of Biomedical Engineering, Faculty of Engineering, Hong Kong Polytechnic University, Kowloon, Hong Kong, China; ^3^School of Biological Science and Medical Engineering, Southeast University, Nanjing, Jiangsu, China; ^4^Department of Orthopaedics and Traumatology, Li Ka Shing Faculty of Medicine, University of Hong Kong, Pokfulam, Hong Kong, China

## Abstract

Cartilage-bone interface (CBI) is a complex structure which bears important information in pathophysiology of osteoarthritis (OA). While high-frequency ultrasound (US) has been widely used for the investigation of articular cartilage, 3D imaging of CBI using US is less commonly reported in this field. Here, we adopted a 3D high-frequency ultrasound imaging approach specifically for the investigation of CBI in human knee samples. Fifteen osteochondral disks from the tibial plateau of seven OA patients were prepared in vitro and scanned using both high-frequency US and micro-CT imaging. The 3D morphology of the tidemark was reconstructed and compared using an image registration approach between the two imaging modalities. Results showed that the 3D tidemark could be well registered between the two imaging methods with a mean surface discrepancy of 33.2 ± 9.9 *μ*m. Quantitative surface waviness/roughness parameter analysis showed significant correlations between the two imaging modalities. An intensity projected en face imaging was proposed to probe characteristic details of the CBI such as its perforations. This study provided evidence for the 3D high-frequency ultrasound as a nonionizing radiation imaging tool potentially useful to evaluate the change of CBI in basic research of join diseases including OA.

## 1. Introduction

Osteoarthritis (OA) is a prevalent chronic joint disease which affects millions of people around the world, especially the aged population [1]. A large proportion of OA-related research focuses on the noncalcified cartilage (NCC), because one hallmark symptom involved in OA is a significant loss of articular cartilage with disease progression. Popular OA grading scales such as the Mankin [2] and the OARSI system [3] heavily rely on the observation of cartilaginous features and treat the cartilage-bone interface change as one of the late-stage OA symptoms. However, OA is a complex disease which involves several different tissues in joint. The subchondral bone (SCB), although less studied compared to cartilage, has also been recognized as an important player in the initiation and progression of OA [4–6] and even leads in OA development before the macroscopic loss of cartilage in certain circumstances [7]. Understanding of SCB and NCC at their interface would provide us a new insight into the pathophysiology of OA at its early stage.

In hyaline cartilage, the calcified cartilage zone (CCZ) is a sandwich layer separated from NCC by an interface called tidemark and from SCB by another interface named the cement line. The role of this layer is twofold serving as a smooth transition for the mechanical loading and providing a crosstalk channel for solute transportation [8]. CCZ mechanically behaves like a matching layer between NCC and SCB so that the whole osteochondral unit is more capable of mechanical loading, as evidenced by tissue-engineered scaffold bearing higher capacities in compressive and shear loading when it is made with a calcified zone than without [9]. A delicate homeostasis is established between NCC and SCB through vascular or other channels in the CCZ, and this homeostasis is broken in OA [10]. Therefore, the change of CCZ including the tidemark bears important information related to the health of the whole cartilage-bone unit. There is a need to develop imaging methods to investigate the change of the cartilage-bone interface (CBI) especially the tidemark for basic research of joint diseases including OA.

Clinically, OA is mainly diagnosed by X-ray radiography where a narrowing of the joint space is typically observed. Various grading systems were proposed to classify the severity of OA such as the International Knee Documentation Committee (IKDC) system for knee joint [11]. However, these clinical systems are not sensitive enough to observe early OA changes, and therefore, imaging methods capable of early OA detection are still demanded. Ultrasound (US), especially high-frequency (>20 MHz) US, has been very early adopted and widely investigated for the imaging of the articular cartilage in previous studies [12]. Ultrasound was firstly introduced in the early 1980s' to measure the thickness and the anatomical distribution of cartilage with verification from other methods [13–15]. Later, various acoustic parameters including speed of sound, backscatter, and reflection coefficients were proposed for tissue characterization in normal and OA cartilage samples [16–21]. Combined with an indentation technique, it became possible to obtain the mechanical properties of cartilage using ultrasound measurement [22–25]. Therefore, comprehensive studies including simultaneous measurement of acoustic, morphological, and mechanical properties can be realized in cartilage using high-frequency US imaging [26], which showed their potential value in the clinical diagnosis of cartilage lesion severity [27]. Although quantitative US parameters such as the integrated reflection coefficient and roughness have been adopted to study the change of CBI in OA [28, 29], there is a scarcity of data in the literature concerning the validation of US imaging in studying CBI. Histomorphometric analysis is a gold method to investigate the CCZ and its surface properties [30]. However, it is too time-consuming concerning a dense sectioning of stained osteochondral tissue for 3D volumetric analysis. Microcomputed tomography (micro-CT) is another capable imaging modality for studying 3D calcified tissue and is recently adopted for the volumetric study of CCZ in OA [31]. The surface of CCZ, i.e., the tidemark, can be extracted from micro-CT data for calculation of quantitative parameters including the roughness.

The CCZ layer is composed of more inorganic material including hydroxyapatite [32], and the stiffness of CCZ is much larger than that of NCC [33]; therefore, it is generally assumed that the second reflection peak in US imaging of osteochondral unit comes from the tidemark, which was indirectly validated by a thickness measurement [14]. In this study, we tried to validate the 3D high-frequency US imaging of CBI using micro-CT imaging. The 3D surface of the tidemark was reconstructed in US imaging and compared to micro-CT imaging using a rigid registration technique. The registration error was computed to evaluate the difference of the two imaging modalities. Macroscopic and microscopic tidemark roughness was also computed and compared for the two imaging methods. Furthermore, an en face projection imaging of the CBI was proposed to observe the microstructure through different depths of the CBI, which could serve as a new tool for investigation of the microstructural change in basic research of OA.

## 2. Materials and Methods

### 2.1. Sample Preparation

Osteochondral samples were collected from the lateral side of the tibial plateau of 7 patients (3 men, 4 women, mean age of 69.4 ± 13.0 years) who received total knee replacement surgery in Queen Mary Hospital (Hong Kong) because of late-stage knee OA. As previously reported, two to three osteochondral disks of 10 mm in diameter were drilled from each sample (Figure 1), and a total of 15 disks were prepared for this study [28]. We purposely obtained these osteochondral disks from the central half of the lateral tibial plateau of OA knees, with less or no articular surface disruption or cartilage worn-out compared to the medial compartment. These osteochondral disks represented an early stage of OA when articular cartilage was less damaged. The samples were preserved in a refrigerator at −80°C and then processed for the 3D ultrasound scanning, micro-CT, and histologic examinations sequentially. A metal pin was inserted into the subchondral cancellous bone from the side of the osteochondral disks for alignment of US and micro-CT imaging. This study was approved by the institutional ethics committee (ref no: UW-09368), and informed consent was obtained from each patient before sample collection.

### 2.2. Ultrasound and Micro-CT Imaging

Disks were transferred from the −80°C refrigerator to a 4°C refrigerator and thawed overnight before the experimental day. At the experimental day, disks were further immersed in physiologic saline solution for at least half an hour to become room temperature before US scanning. The disk was then fixed with plastic clay (BluTack, Bostik, Thomastown, Australia) at the bottom of a container for 3D US scan (Figure 2). B-mode US image sequences were collected using a linear array transducer (MS550D, VisualSonics Inc., Toronto, ON, Canada) of a high-frequency ultrasound imaging system (Vevo LAZR, VisualSonics Inc., Toronto, ON, Canada). The −3 dB bandwidth of the US transducer was 17–33 MHz with a central frequency of 25 MHz. The axial resolution and lateral resolution were about 40 *μ*m and 80 *μ*m according to specifications provided by the manufacturer. The transducer was fixed in a platform which could be translated in one direction (*y* in Figure 2), and its azimuth direction was set in a perpendicular direction (*x* in Figure 2) to acquire 3D US image sequences of the tested disk. The *y*-scan followed the direction of the metal pin inserted in the disk. A square region with a side length of 7 mm was scanned for each disk, i.e., the width of each B-scan image was 7 mm in the *x*-direction and the linear stage moved for another 7 mm in the *y*-direction. The depth coverage was 7 mm which was enough to scan the whole depth of the cartilage and the CCZ region. Because of strong reflection from CBI, the deep part of the subchondral bone appeared dark below a small bright region near the tidemark (see typical US images in Figure 3). Its step size was set to be 32 *μ*m, and therefore a total of 220 B-scan images were collected from one disk. The pixel size was 15 *μ*m × 15 *μ*m in the “*xz*” plane for each B-scan image. During the experiment, a single focus was set, and the focal point was placed approximately at the position of tidemark, i.e., the second bright line in the US image. The disk orientation was adjusted to obtain a maximally reflected signal from the tidemark before data collection, indicating an optimized perpendicularity between the US beam and the tidemark. After a proper position was configured for the tested disk, data acquisition was started and B-scan sequential images were collected and saved for offline analysis, which is described in details in the next subsection.

Micro-CT imaging was performed after US imaging for assessing the subchondral bone quality and quantity using similar protocols reported in a previous study [34]. In brief, a micro-CT system (VivaCT 40, Scanco Medical AG, Bruttisellen, Switzerland) with a tube voltage of 70 kVp, tube content of 0.114 mA, and an isotropic voxel scan size of 21 *μ*m × 21 *μ*m × 21 *μ*m was used for imaging of the prepared disks. The whole 3D bone structures were generated, and its quality could be quantitatively analyzed via the associated micro-CT software (Scanco Medical AG) including bone mineral density (BMD) and bone volume fraction (BV/TV). For direct comparison with the US imaging in this study, micro-CT images (~500 pictures for each disk) were exported from the micro-CT system and saved for offline analysis which is also detailedly described in the next subsection. After micro-CT scanning, the samples were decalcified, sectioned in thin slices, and embedded in wax sequentially for routine histopathologic examination (Safranin O and fast green staining), using our established protocols [34].

### 2.3. Image Processing and Data Analysis

#### 2.3.1. Extraction of 3D Tidemark Surfaces from US and Micro-CT Images

US images were firstly processed by a semiautomatic procedure of tidemark segmentation. An approximate surface profile was manually drawn in an open-source software (ITK-SNAP, ver. 3.8.0-beta, http://www.itksnap.org/) [35], and the position of which was read in custom-written codes of Matlab (ver.2017b, Mathworks Inc., Natick, MA, USA) for extraction of the true tidemark surface. For simplicity, tidemark surface was found from each vertical line along the horizontal direction by searching the first peak reflection above a noise level in a window of 20 pixels (~0.30 mm) centered at the manually drawn surface profile point. The noise level was calculated as the reference signal in the saline solution, i.e., the dark part on the top before the cartilage surface. As there might be some small cracks in the tidemark, a dark zone indicating a broken tidemark might exist in the US imaging. If no peak signal was detected in this case, this line was considered as a crack, and the tidemark point was obtained by interpolation from its neighbor tidemark points. Then, a 2D tidemark profile (*xz* plane in Figure 2) was extracted from each image, and all the surface profiles in sequence constructed a 3D tidemark surface profile, which would be compared to that of micro-CT imaging (Figure 3).

For the micro-CT images, they were rotated firstly by a small angle to place the tidemark surface in an approximately horizontal direction by evaluating the surface level of the volumetrically averaged image of a scanned disk. Then, they were processed by an Otsu thresholding [36] and binarization to obtain the calcified tissue with high contrast. The extraction of the tidemark surface point was similar to that of the ultrasound image. The tidemark surface point was found by detecting the first abrupt change in each vertical line. When no surface point was detected because of holes or cracks, two neighbor surface points were found, and a smooth line was filled in between by interpolation. All the surface profiles found from each micro-CT image were reconstructed as a 3D surface of the tidemark (Figure 3).

#### 2.3.2. Quantitative Comparison of 3D Tidemark Surface from US and Micro-CT Images

Tidemark surfaces reconstructed from the US and micro-CT imaging were compared, and their degree of correspondence was evaluated through image registration. An averaged distance discrepancy was used to indicate the difference between the registered two tidemark surfaces from the two imaging modalities, which is defined as follows:

(1) $$\begin{array}{c} D_{diff}=\frac{1}{N}\overset{N}{\underset{i=1}{\sum }}\left(d\left(p_{US,i},s_{mCT}\right)\right) \end{array}$$

where *d*(*p*_*US*,*i*_, *s*_*mCT*_) is the distance from the tidemark surface point *i* in the US imaging to the reference surface *s*_*mCT*_ in the micro-CT imaging. The image registration and average distance discrepancy computation were performed using free software CC (CloudCompare, ver. 2.10.2, https://www.danielgm.net/cc/). The core technique used in the registration is the iterative closest point (ICP) searching algorithm with an optimized rigid transformation combining both translation and rotation [37]. ICP is the most popular algorithm to register two 3D point clouds with no need to know the correspondent point sets. In registration, an error difference of 0.01 *μ*m between two iterations was set as a threshold to stop the iteration. After registration, an average distance between a target surface (US imaging in this study) and a reference surface (micro-CT imaging) could be calculated automatically, which was treated as the average discrepancy *D*_*diff*_ between the 3D US/micro-CT imaging of tidemark.

Furthermore, quantitative surface morphological parameters including the surface waviness (macroscopic surface smoothness, SW) and roughness (microscopic surface smoothness, SR) were also calculated from the extracted surface profiles in US and micro-CT imaging. In detail, a mean (*S*_*a*_) and root mean square (RMS) (*S*_*q*_) surface topology variation index was computed from the surface profile for SW and SR, respectively, which are defined as follows:

(2) $$\begin{array}{c} S_{a}=\frac{1}{MN}\underset{i,j}{\sum }\left|s_{i,j}-{SR}_{i,j}\right| \end{array}$$

(3) $$\begin{array}{c} S_{q}=\sqrt{\frac{1}{MN}\underset{i,j}{\sum }{\left(s_{i,j}-{SR}_{i,j}\right)}^{2}} \end{array}$$

where *i*, *j* indicate the digitalized location index in the *x*-*y* scan plane, *M*, *N* are the total number of scanned locations in each direction, *s* is the extracted surface position in the *z* direction, and *SR* is the macroscopic/microscopic reference surface in calculation of SW/SR. For waviness, *SR* is a reference surface obtained by fitting a first-order (counting for tilts of *x* and *y*) flat surface for the whole 3D surface profile; for roughness, *SR* is a reference surface including the surface waviness which is obtained by fitting a higher-order polynomial (for *x* and *y*) surface for the whole 3D surface profile. The reference surface in calculating waviness/roughness was obtained using the Matlab function “fit” with controlled parameters of “poly11”/“poly55”, where “1”/“5” indicates the highest order used in the polynomial curve fitting. The relationship between the surface parameters of the US/micro-CT was analyzed using the Pearson correlation (*r*). A level of *p* < 0.05 was considered to have a significant correlation. It should be noted that waviness and roughness indices were independent parameters for each disk. An osteochondral disk with a large value of waviness might not necessarily have a large value of roughness and vice versa.

#### 2.3.3. Qualitative Comparison of CBI Region from US and Micro-CT Imaging

For both US imaging and micro-CT imaging, an en face imaging is adopted to observe the change of different morphologies of CBI along the depth direction (Figure 3). En face imaging is a viewing technique used to generate a 2D projection image from the depth direction, which has become very popular in the field of ophthalmic imaging, particularly for viewing photoreceptors and vascular network of the posterior eye [38]. This imaging method could be used here to observe typical structures of the CBI including perforations or channels in the calcified/bony structure. Different thickness of CBI could be included in en face imaging to show the variation of structures along the depth. Maximal intensity projection (MIP) and average intensity projection (AIP) could be used to generate the en face images for observing similarity and difference between the two imaging modalities.

## 3. Results

### 3.1. Surface Registration Analysis

All the tidemark surfaces were successfully reconstructed in US and micro-CT imaging. 3D surface registration could be achieved typically in several to ten minutes using a PC installed with an Intel i7 4-core CPU and 16GB RAM. The process could be accelerated by a manual coarse alignment of the two surfaces before ICP registration. A good registration could be also confirmed by comparing the metal pin observed in micro-CT with the reference scan direction in US. Typical results of comparison of the two surfaces after ICP registration are shown in Figure 4. For each scanned disk, an averaged distance and its standard deviation were obtained using the cloud/mesh distance computation tool provided by CC. Then, this distance was averaged for all the studied 15 disks. An overall value of 33.2 ± 9.9*μ*m (range, 20.8-55.8 *μ*m) was obtained as an averaged distance discrepancy between the two tidemark surfaces from the US/micro-CT imaging after registration.

### 3.2. Surface Roughness Analysis

Quantitative surface parameters including waviness (SW) and roughness (SR) were calculated for each disk.  Figure 5 shows typical results of a 3D view of tidemark surfaces with relatively small and large values of the SW/SR index. Corresponding histology results also confirmed the roughness difference between the two samples (Figure 6). The Pearson correlation analysis is presented in Table 1. It was found that SW/SR indices had a significant correlation between the two imaging modalities (*p* < 0.05, refer to the column-wise correlation analysis in Table 1), while there was no significant correlation between SW and SR for both the US and micro-CT imaging (*p* > 0.05, refer to the row-wise correlation analysis in Table 1). A further correlation analysis was conducted between the surface discrepancy of the two imaging modalities and the SW/SR, but no significant correlation was found (*p* > 0.05). It was noted that the SW/SR index was generally larger in the micro-CT than US imaging.

### 3.3. En Face Imaging

A tissue volume of interest (VOI) with different thickness (from 1 pixel to ~10 pixels, i.e., from ~20 to ~150 *μ*m) was used for en face imaging and typical results of MIP en face imaging are shown in Figure 7. For US en face images, large regional grayscale variation was observed such as the brighter region observed in the left part of the image compared to the darker one on the right (Figure 7(a)), which might be due to the signal intensity variation induced by change of acoustic beam incidence angle because of macroscopic surface profile change. In small regions, a typical texture pattern consisting of thin dark channels forming interconnected loops similar to the capillary vascular network was observed for all disks, for which the possible explanation in correspondence with tissue structure and physiology is presented in the Discussion part. Dark vertical stripes as image processing artefacts were observed in all disks when a thin tissue region was included (*T* = 15 *μ*m thickness case in Figure 7(a)), which might be due to inconsistency of reference line drawing in consequent image frames. When the tissue VOI thickness increased, this artefact became smaller and almost vanished for tissue thickness of *T* = 150 *μ*m. For micro-CT imaging, the porosity of the CBI was observed as small dark holes with the varied size of diameters in the en face images (Figure 7(b)), which might show direct channels for material exchange between bone and cartilage. The micro-CT images appeared more homogeneous or “clearer” than the US images. The signal became brighter along with the increase of thickness included in MIP en face imaging (Figure 7(b)). Overall, the texture of the en face US images of the CBI appeared grainier and its intensity varied in a larger extent than that of the micro-CT images. The AIP en face images (not shown) were similar to the MIP (shown in Figure 7), excluding a general decrease of the overall intensity under the same thickness of VOI because of averaging. The vertical stripe effect in US was more obvious in AIP than in MIP.

## 4. Discussion

This study aims to propose a 3D high-frequency US imaging method to investigate the articular cartilage-bone interface (CBI), particularly the tidemark morphology, with validation results from the micro-CT imaging. Results showed the 3D tidemark surface could be successfully extracted from the US imaging with a good correspondence from micro-CT imaging, in terms of surface profile and smoothness (waviness/roughness). However, en face imaging showed quite different appearance of the CBI region in the US and micro-CT imaging. These observations demonstrate US imaging is potentially a viable and unique tool in future study to probe CBI and its role in early development of OA.

In this study, B-scan images were used for the imaging of CBI because the pixel resolution (15 *μ*m) was already comparable to that of the micro-CT (21 *μ*m). Radiofrequency-based A-line signal and analysis technique can be adopted if better resolution or regression along depth for extraction of acoustic parameters such as attenuation is needed [17]. The tidemark was detected by a semiautomatic segmentation of NCC-CCZ interface, which was realized by searching the peak of the reflected US signal near the manually drawn tidemark boundary. This segmentation scheme was reasonable because of a significant change of the acoustic impedance along the tidemark, which would result in a large reflection [14, 28]. Several factors would affect the accuracy of the tidemark detection, which includes the insonation angle, speed of sound, and tissue preparation procedure [39]. The insonation angle was adjusted in our study to obtain an optimally reflected signal from the CBI, and therefore the image was optimal in terms of the signal quality. A precise tidemark position computation in the US measurement depended on the selected speed of sound in its propagation in cartilage, which was not specifically obtained in the current study. A recent study showed that a predefined adjustment of the speed of sound from 1580 m/s to 1696 m/s did not result in improvement of cartilage thickness measurement, which might be due to a large variation of speed of sound in articular cartilage with respect to the anatomical sites, composition and degeneration states [39]. Therefore, this simple way of correction using a direct adjustment of speed of sound seems not effective to improve the detection accuracy and was not adopted in this study. A significant difference of speed of sound is known between the uncalcified cartilage and the calcified cartilage; however, this would not affect the extraction of the tidemark because the tidemark was on the top of the calcified cartilage. For the preparation procedure, the osteochondral disk was not fixed but was kept in the physiologic saline solution in US and before micro-CT imaging, so a minimal effect was assumed for the change of CBI between the US and micro-CT imaging so direct comparison could be performed.

While it is known the histomorphometric analysis is an ideal method to study CBI [30], this technique is too complex and time-consuming to be practical for clinical use. Micro-CT is an alternative and recently has been demonstrated to be an effective approach to study the topological change of tidemark and the perforation in CCZ [31]. Micro-CT was used as a reference method to extract the 3D tidemark surface in this study. The 3D tidemark surface was detected by searching the abrupt change between NCC and CCZ in micro-CT images. This processing was quite straightforward except when a small number of noncalcified vascular or soft tissue channels (dark holes) were detected in the processing. In this case, the gap was filled with a regressed line between its neighborhood interface points. This might bring some uncertainty of accuracy when compared to US, in which these channels might not be obviously seen correspondingly. Tidemark surfaces obtained from US and micro-CT were compared using a 3D registration approach. Comparison using the 3D registration had the advantages of no need to specifically consider the position alignment required in 2D imaging, which improves the reliability of our results. Bearing the accuracy concerning factors discussed so far in mind, we found an average discrepancy of 33.2 ± 9.9 *μ*m for the two 3D tidemark surfaces after registration, which shows a good agreement between the two imaging modalities. The discrepancy might come from the abovementioned factors in the measurement procedures as well as the intrinsic difference of image contrast in the two imaging modalities. Tidemark surface from the US imaging is based on the significant change of acoustic impedance beside this interface, while it is the contrast of X-ray attenuation in the micro-CT imaging. There might be some difference between the position of significant change in acoustic impedance and that in X-ray attenuation near the tidemark, although small, thus creating the two-surface discrepancy, which warrants further investigation.

Among various morphological parameters, the roughness of the tidemark is an important parameter which could be used to characterize OA development [28, 31]. A waviness/roughness (SW/SR) index which reflects the macroscopic/microscopic smoothness of the tidemark is defined in this study. A significant correlation was found for these parameters obtained between the US and micro-CT imaging. The waviness is a parameter reflecting the anatomic change of the surface topology while the roughness reflects more local change, and therefore the latter may be more practically useful in characterizing disease development. The waviness was significantly larger than the roughness (Table 1) for the studied disks, which showed the tidemark surfaces varied in a larger range because of the anatomic change of surface topology. A larger waviness/roughness value was found in the micro-CT than the US which might be due to a noncalibrated distance scale for the two imaging modalities. Wang et al. found that the cement line under the bottom of CCZ had a larger roughness than that of the tidemark which might also be significantly affected in early OA development [30]. Unfortunately, the cement line is not directly observable in both imaging methods due to a small contrast for either acoustic impedance or X-ray attenuation near this boundary. In general, micro-CT is also limited in detecting the cartilage layer but recent studies showed that contrast agents such as phosphotungstic acid could be used in micro-CT to enhance the visibility of both the cartilaginous layer and the tidemark in basic research of OA [40, 41]. Therefore, contrast-enhanced micro-CT might be considered in future investigation which could provide a more precise 3D morphology of the CBI as a reference for ultrasound imaging.

An en face imaging mode was proposed in this study to show the projected image of the CBI layer with different thickness. In US, the en face image showed regional variation of brightness, most probably because of insonation angle change for different parts of the surface. This phenomenon was not observed in micro-CT imaging because the quality of micro-CT was independent on positioning of the scanned sample. Perforations of the CBI were observed in the micro-CT imaging which might be the channels of either vasculature or soft tissues. This was consistent with previous studies demonstrating direct connection between NCC and subchondral bone for exchange of nutrition and metabolites through these channels [31, 42]. This pattern of perforation was not typically observed in en face image of US imaging. As the horizontal resolution of the US imaging used in this study was ~80 *μ*m, which was larger or comparable to the perforation size, those channels seemed not clearly resolved in the US imaging. However, a detailed analysis shows that US imaging could also indicate some echolucent regions breaking through the CBI, which might be perforations in the CCZ and the subchondral bone (Figure 8). Furthermore, interconnected echolucent channel network was found typical in the US en face images which might indicate there were channels in the CBI, and these channels were interconnected similar to microvascular network. Unfortunately, these observations were not confirmed by reference imaging method in the current study. The potential of US imaging in detecting perforations (porosity) or even their interconnected network of the CBI needs to be further investigated. Currently, this method cannot be directly applied to in vivo situations but further development of a miniaturized arthroscopic probe may realize a straightforward application of the current assessment method.

In summary, high-frequency ultrasound was utilized for the 3D imaging of the cartilage-bone interface, with results compared to the micro-CT in this study. The 3D tidemark surface showed a small discrepancy between the two imaging modalities after registration. Significant correlations were found between the two imaging methods for the waviness/roughness surface smoothness parameters. En face imaging of the cartilage-bone interface region in the ultrasound imaging showed quite specific texture pattern compared to the micro-CT imaging, which might reflect characteristic structure in the calcified cartilage zone. Our study demonstrated that high-frequency ultrasound is a potential method to investigate the 3D topological change of tidemark and the structural variation of the cartilage-bone interface region in future research of joint disease pathophysiology such as osteoarthritis.

## Figures and Tables

**Figure 1:** A schematic drawing showing extraction of osteochondral disks of 10 mm in diameter from the lateral tibial plateau in this study.

**Figure 2:** A schematic showing the US imaging setup. Multiple US images were collected by translating the US transducer along a linear stage. Refer to text for detailed procedure.

**Figure 3:** A schematic showing the processing of ultrasound and micro-CT imaging data to obtain a 3D tidemark surface and en face imaging of the cartilage-bone interface. 3D surface is obtained by connecting all the surface lines extracted from each ultrasound/micro-CT image in scan sequences. En face image is obtained by projecting data in a certain thickness region beyond the tidemark.

**Figure 4:** (a) Registration of two tidemark surfaces obtained from the ultrasound (gray) and micro-CT (green) imaging. The white arrow shows the direction of the inserted metal pin. (b) Clouds/mesh distance mapping for ultrasound obtained tidemark surface to that from micro-CT after registration. Shown on the right is the color bar used for distance mapping in unit of mm. An averaged distance discrepancy of 26.8 ± 22.9 *μ*m (mean ± SD) was obtained in this case.

**Figure 5:** (a) 3D view of two typical tidemark surfaces with a small and large waviness index (*SW*_*a*_ = 50.4*μ*m and *SW*_*a*_ = 178*μ*m, respectively). (b) 3D view of two typical tidemark surfaces with a small and large roughness index (*SR*_*a*_ = 22 *μ*m and *SR*_*a*_ = 36*μ*m, respectively). A scale color bar in unit of mm is shown for the height mapping.

**Figure 6:** Comparison of typical cross-sectional images in the ultrasound imaging and histology (Safranin O staining) for two specific samples with a small and large roughness index as shown in Figure 5(b). (a, c) Represent a typical US and histology image for the sample with a roughness index of *SR*_*a*_ = 22 *μ*m; (b, d) represent a typical US and histology image for the sample with a roughness index of *SR*_*a*_ = 36 *μ*m. The results consistently show a smoother surface in (a) and (c) compared to those of (b) and (d) in terms of US imaging and histology. Duplicated tidemark obviously seen in histology (c) is also implicitly observed as a second bright reflection surface in US imaging (a). The scale bar is 1 mm in length.

**Figure 7:** Typical en face images for the ultrasound and micro-CT imaging. (a) MIP images of the ultrasound imaging with different VOI thickness: 15, 45, 105, and 150 *μ*m, respectively. (b) MIP images of the micro-CT imaging with different VOI thickness: 21, 42, 105, and 147 *μ*m, respectively. The ultrasound scanning direction (arrow) is indicated in the last images of (a) and (b) for the reference of comparison. The rectangular box in (b) indicates the region of ultrasound imaging. The scale bar is 1 mm in length.

**Figure 8:** A detailed analysis of a US en face image (left) with two specific cross-sectional B-images (right) shown on two positions as indicated by the two dotted lines. Arrows (1 and 2) show two typical echolucent regions in the en face image and also correspondingly in B-mode images, which might indicate perforations in the CBI. Scale bar shows 1 mm in length.

**Table 1:** Measured waviness/roughness index and correlation analysis from US and micro-CT imaging.

	Waviness (*μ*m)		Roughness (*μ*m)		*r* (*p*)
Modalities	*SW*_*a*_	*SW*_*q*_	*SR*_*a*_	*SR*_*q*_	
US					
*S*_*a*_	113 ± 52		33 ± 9		0.07 (0.80)
*S*_*q*_		146 ± 65		47 ± 21	0.13 (0.64)
Micro-CT					
*S*_*a*_	160 ± 52		44 ± 13		-0.46 (0.09)
*S*_*q*_		205 ± 63		66 ± 30	-0.22 (0.42)
*r* (*p*)	0.90^∗^ (<0.001)	0.90^∗^ (<0.001)	0.77^∗^ (<0.001)	0.82^∗^ (<0.001)	

*S*_*a*_: absolute mean index; *S*_*q*_: root mean square (RMS) index (refer to the text for definitions); *SW*: waviness; *SR*: roughness; *r*: Pearson correlation, *p*: significance level of Pearson correlation analysis. ∗: significant correlation (*p* < 0.001).

## Data Availability

The extracted 3D surface data files in ‘stl' format from US and micro-CT imaging used to support the findings of this study have been deposited in the ‘Dropbox' cloud platform. These and other related data are available from the corresponding author upon request.
